This article has been retracted.

# Alleviation of temperature stress in maize by integration of foliar applied growth promoting substances and sowing dates

**DOI:** 10.1371/journal.pone.0260916

**Published:** 2022-01-20

**Authors:** Irfan Afzal, Shakeel Imran, Talha Javed, Ayesha Tahir, Muhammad Kamran, Qamar Shakeel, Khalid Mehmood, Hayssam M. Ali, Manzer H. Siddiqui

**Affiliations:** 1 Seed Physiology Lab, Department of Agronomy University of Agriculture, Faisalabad, Pakistan; 2 Department of Agronomy, University of Agriculture, Vehari, Pakistan; 3 College of Agriculture, Fujian Agriculture and Forestry University, Fuzhou, China; 4 Fodder Research Sub-Station, Ayub Agricultural Research Institute, Faisalabad, Pakistan; 5 Rothamsted Research Institute, North Wyke, Oakhampton, Devonshire, England; 6 Department of Botany and Microbiology, College of Science, King Saud University, Riyadh, Saudi Arabia; Anhui Agricultural University, CHINA

## Abstract

Temperature is a key factor influencing plant growth and productivity, but its sudden rise can cause severe consequences on crop performances. Early sowing and application of growth promoting agents as a foliar spray can be a sustainable approach to cope with high temperature stress at grain filling stage of cereal crops. Therefore, a test was designed to explore the potential of different growth helping agents including sorghum water extract (SWE, 10 ml L^-1^), moringa leaf extract (MLE, 3%), hydrogen peroxide (H_2_O_2_, 2 μM), salicylic acid (SA, 50 mg L^-1^) and ascorbic acid (ASA, 50 mg L^-1^) as foliar agents at different sowing dates (early and optimum) to cope with temperature stress in maize. The results stated that foliar application of growth promoting substances successfully persuaded high temperature tolerance at reproductive phase of maize in early and optimum sowings when compared to control. However, SWE + ASA, MLE + H_2_O_2_ and SWE + ASA + SA + H_2_O_2_ were the best combinations for improving growth, development, and physiological variables under both sowing dates even under suboptimal temperature. All foliar applications significantly increased maize grain and biological yields while maximum was observed in SWE + ASA followed by SWE + ASA + SA + H_2_O_2_ or MLE + H_2_O_2_ that were statistically at par with ASA + SA + H_2_O_2_ but plants without spray or distilled water application did not improve grain and biological yields. Overall, the foliar applications of growth promoting substances enable the plant to enhance its growth, development, morphology, yield and biochemical variables.

## 1. Introduction

Maize (*Zea mays*) is one of the world’s three major staple crops, with wheat and rice, and is geographically the most widespread of the three with approximately 50–60% contribution of per day human energy requirements, feed for livestock and raw material for industry [1]. Maize plays a pivotal role because of its high nutritional profile, availability of excess amount of micronutrients like abundant quantity of macronutrients such as fiber, starch, fats and fiber, proteins and fat alongside micronutrients like ß-carotene, B-complex vitamins, ß-carotene and essential minerals i.e., phosphorus magnesium, copper and zinc, and [2]. Maize is sown two times a year i.e., autumn and spring seasons, in Pakistan [3]. The spring crop shows more potential and yield when compared to autumn crop. However, increased temperatures at the time of anthesis severely retard the yield potential of the crop [4]. Temperature above 38°C during seed development results in pollen desiccation, poor seed setting, and smaller grains by elevating grain filling duration and ultimately lower seed yield [5]. High temperature during reproductive phase is becoming a major area of concern for affecting crop production and productivity worldwide. Higher temperatures lead to induce cellular stress which becomes the reason for the overproduction of reactive oxygen species (ROS) which damages nucleic acids, proteins and lipids eventually consequential cell death [6]. In addition to temperature stress the drought conditions faced by the maize crop results in a decreased kernel set [7]. The damage caused by heating becomes more severe with the creation of ROS [8]. This formation of ROS becomes the reason of oxidative damages in different cell structures and macromolecules along with the limitations in essential nutrient uptake such as potassium [9]. Adaptation of early sowing for spring crop of maize can be beneficial in avoiding the lethal heating periods at the time of anthesis and maturity. Although, the early sowing for spring maize helps in preventing the heat injuries but the exposure of low temperatures (below 10°C) becomes the reason of slower imbibition rates and poor germination [10].

Exogenous application of synthetic and organic compounds like antioxidants, osmo-protectants and plant growth regulators is a valuable technique to lessen the undesirable effects of environmental stressors on different crops [11]. Several important growth promoting substances like salicylic acid (SA), moringa leaf extract (MLE), H_2_O_2,_ ascorbic acid (ASA) and sorghum water extract (SWE) and have been proved beneficial to lower both the heating and chilling injuries on the developmental and yield characteristics of the crops. These growth promoting substances lowers the formation of reactive oxygen species and slows down the senescence in maize [12]. Plant growth and physiological attributes are evidently improved when using the 3% MLE solution as a foliar spray to the plant at its growing stage, even under harsh conditions [13]. Exogenous application of MLE improved chlorophyll contents, total phenolics, antioxidants, leaf area, grain weight and yield of wheat grown in stressful conditions [14, 15]. Exogenous applications of growth promoting compounds i.e., ASA, SA and H_2_O_2_ as spraying agents are also reported to regulate the plant’s reaction to resist unfavorable effects of temperatures on development and kernel production of maize [16–19].

Previously, efficacy of naturally occurring plant growth promoting agents such as MLE and SWE alone or in combination with synthetic growth promoting substances against temperature stress were explored under lab conditions [18]. Therefore, it is vital to investigate the potential of naturally occurring and artificial growth promoters as foliar spraying agents during important stages of growth at field level. Thereby, this study aims to investigate the effect of foliar applied natural growth promoting agents such as MLE and SWE along with the combinations of other synthetic growth promoters against heat stress during growth and developmental phases through modulation of physiological and biochemical processes.

## 2. Materials and methods

### 2.1. Crop husbandry

Field experiment was conducted at Research area, Department of Agronomy, University of Agriculture, Faisalabad City, Punjab Province, Pakistan (30.37° N, 69.34° E) during the months of January-June 2011. The experiment was laid out in randomized complete block design (RCBD) with split plot arrangement, randomizing the sowing dates in main plots and foliar applications in subplots with four replications. Single cross hybrid spring maize cv. Pioneer 32F10 with 96% capacity for germination was brought in from Pioneer Seeds, Sahiwal, Pakistan (30.6682° N, 73.1114° E) and utilized for the experimental purpose. The initial quality parameter is including the moisture content of seeds and the seed lot’s physical purity was 12.5% and 99.90%, respectively. The textural class of the soil was non-sandy that had a pH (7.3), EC (0.413 dSm^-1^), phosphorus available (13.02 ppm) the level of potassium (365.61 ppm). The net size of the plot was maintained at 2.00 m x 3.75 m.

The seeds of maize were sown in the early phase (January 15, 2011) and the best (February 15, 2011) dates for sowing. The distance between the plants was kept at 75 cm apart in rows, at different dates of sowing, two seeds were dibbled at 25 cm apart holes. The NPK @ 200, 100 and 100 as Urea, Diammonium phosphate (DAP) and Sulphate of Potash (SOP) were used as fertilizers during the course of the study. Half of the total dose of nitrogen was applied at sowing time, whereas the remaining half dose of nitrogen was applied with the first irrigation. All other agronomic and plant protection practices were remained uniform for all treatments.

### 2.2. Growth promoting substances

Leaves of moringa and sorghum were harvested from fully matured plants, after extraction with locally assembled machine, respective solutions were prepared for experimental purpose. The solutions of synthetic growth promoting agents were prepared based on active ingredients and purity percentages. The synthetic growth supporting materials were bought from Merck, Germany. The growth promoting agents used were sorghum water extract (SWE, 10 ml L^-1^), moringa leaf extract (MLE, 3%), hydrogen peroxide (H_2_O_2_, 2 μM), salicylic acid (SA, 50 mg L^-1^) and ascorbic acid (ASA, 50 mg L^-1^). The experimental units were sprayed with the agents utilized at crucial growth times (height of knee, tasseling and development of grain) of the maize crop. The treatments applied were as mentioned; 3 distilled water spray, SWE+H_2_O_2_, MLE+H_2_O_2_, ASA+SA+H_2_O_2_, SWE+ASA+SA+H_2_O_2_ and were compared with control (without foliar application).

### 2.3. Growth and development

Five maize plants were selected at random from every experimental unit to calculate the leaves number, leaf length and plant height twice a week. The mean values of leaves per plant, leaf length and plant height were determined. To determine crop growth rate, plants were harvested per square meter, rinsed with water that had been distilled, and their weight was taken while fresh, that was followed by drying in the oven at 65°C till constant weight. After drying, dry weights were recorded and converted to crop growth and net assimilation rates, using the formula according to formula suggested by Reddy [20].

### 2.4. Physiological attributes

Determination of net rate of photosynthesis, stomatal conductance and transpiration was done at anthesis from the top of an expanded third leaf, utilizing a system that was open LCA-4 transportable infrared gas analyzer (ADC BioScientific Ltd., Hoddesdon, UK). The optimum time to record these observations was 09:00 a.m. to 12:00 p.m. with specifications as stated; leaf chamber volume gas flow rate (v) 391 mL min^-1^, surface area of leaf 12.25 cm^2^, ambient pressure (P) 98.89 kPa, leaf chamber molar gas flow rate (U) 249 μ mol S^-1^, leaf chamber’s temperature (Tch) varied from 40.2 to 44.6°C, grinder flow of air per unit area of leaf (Us) 232.16 mol m^-2^ S^-1^, PAR (Q leaf) at surface of leaf was highest up to 921 μ mol m^-2^.

### 2.5. Biochemical analysis

The chlorophyll a and b were defined with the technique as defined by Arnon [21]. About 0.5 cm of fresh leaves segments were cut and extracted overnight in 80% acetone at a temperature of 100°C. The extract was then centrifuged for 5 minutes at 14000 rpm for 5 min and the supernatant was utilized to read the absorbance of supernatant was read at 645 and 663 nm with the help of using a spectrophotometer (T60 U Spectrophotometer, PG Instruments Ltd., Leicestershire, UK). For the determination of total phenolics, leaves were crushed in pestle and mortal by making use of liquid nitrogen. A sample of 20 μl was added to 100 μl Folin-Ciocalteu chemical (2 N), 1.60 mL distilled water, and 300 μl sodium carbonate mixture in a test tube [22]. After 30 min of heating at 40°C in water bath, test tubes were instantly shifted in ice box and absorbance was read at 765 nm by using spectrophotometer (T60 U Spectrophotometer, PG Instruments Ltd., Leicestershire, UK).

The anthrone method was used to determine the total stable sugars present in the samples of leaves. A mixture was prepared by using 5 mL of 2.5 N HCl and using Ground leaf sample (25 mg) in a test tube. Test tubes were heated for 3 hours at 100°C in water bath and then lowered to a normal room temperature Tubes were placed in water bath 100°C for 3 h followed by cooling of tubes at room temperature. Distilled water was added gradually to make the total volume of the tube to 100 mL before centrifugation at 4000 rpm for the period of 10 minutes.0.5 mL supernatant, 0.5 mL distilled water and 4 mL anthrone (0.2% v/v anthrone on 95% sulfuric acid) was taken in another tube. The test tube was heated in boiling water for 8 min and cooled down quickly before taking the reading at 630 nm. The tube was heated again in boiling water bath for 8 minutes. The tube was cooled rapidly, and reading was taken at 630 nm by using spectrophotometer (T60 U Spectrophotometer, PG Instruments Ltd., Leicestershire, UK).

Catalase activity (CAT) was measured with the same method explained by Chance and Maehly [23] with a few modifications. 3 mL of CAT solution was made by adding 15 mM H_2_O_2_, 50 mM phosphate buffer (pH 7.0) and 0.1 mL enzyme extract to start the process of reaction. The change in the absorbance was measured at 240 nm after each 20 seconds that passed. Alterations in absorbance of 0.01 units per 60 second is defined as single-unit CAT action. The activity of enzyme was expressed on a protein basis. Protein strength of extract was measured by Bradford [24]. For 3 mL of POD reaction mixture, 40 mM of H_2_O_2_, 50 mM sodium acetate buffer with 5.0 pH, 20 mM guaiacol and 0.1 mL of enzyme extract was added. Absorbance changes were recorded after every 20 s at 470 nm. Absorbance change of 0.01 units per minutes is known as one-unit POD activity. Protein based activity of each enzyme was expressed and protein concentration was calculated following the method by Bradford [24]. SOD activity was possible to measure because of its ability to impede photochemical reduction of nitroblue tetrazolium (NBT) [25]. For this reaction, the solution mixture requires 50 μM NBT (NBT dissolved in ethanol), 50 μL enzyme extract, 1.3 μM riboflavin, 50 mM phosphate buffer (pH 7.8) and 13 mM methionine, 75 nM EDTA. These elements are mixed to make up to 3 mL of the solution mixture for measuring SOD activity. The reaction mixture was kept in a container allowing 15 W of illumination for 15 min. The absorbance was then measured at 560 nm with the help of spectrophotometer (T60 U Spectrophotometer, PG Instruments Ltd., Leicestershire, UK).

### 2.6. Yield and yield related parameters

Fiver plants were randomly selected from each experimental unit to determine the number of cobs per plant, cob diameter and test weights. Thirty plants were randomly selected from each experimental unit, sun dried and threshed. Grains were separated from straw, weighed on electric balance to get grain yield and biological yield of thirty plants and converted into Mg ha^-1^.

### 2.7. Statistical analysis

The data was analyzed, according to the Fisher’s analysis of technique of variance. The least significant difference at the probability of 5% was utilized so that the treatment means can be compared [21]. Principle component analysis was performed using ‘XLSTAT ver. 2019’.

## 3. Results

### 3.1. Growth and developmental analysis

All foliar applications improved crop growth rate (CGR), however SWE + ASA and MLE + H_2_O_2_ applications were the most considerable in both sowing dates. Minimum CGR was produced by the crop plants of control and distilled water spray (DWS). Dry matter accumulation (DMA) was recorded biweekly, and DMA increased in a linear fashion and attained maximum value at 90 days after sowing (DAS). All foliar applications significantly enhanced DMA in both sowing dates but the performance of MLE + H_2_O_2_ and SWE + ASA was utmost than others (Fig 1). Net assimilation rate (NAR) was peaked at 45–60 DAS then it decreased gradually (Fig 1). Foliar application of MLE + H_2_O_2_ and SWE + ASA + SA + H_2_O_2_ remained most effective followed by SWE + ASA as compared to other treatments including control (Fig 1). Applications of SWE + ASA and SWE + ASA + SA + H_2_O_2_ were found most effective in improving leaves per plant followed by MLE + H_2_O_2_ and ASA + SA + H_2_O_2_. Foliar applications of SWE + ASA and SWE+ ASA + SA + H_2_O_2_ at knee height stage of spring maize hastened the leaf length more effectively as compared to other treatments in both sowing dates (Fig 2). Rather long leaves were observed in early sowing. Furthermore, early sown crop plants achieved more height than optimum planting. Foliar application of SWE + ASA + SA + H_2_O_2_ and ASA + SA + H_2_O_2_ were effective for improving plant height in early sowing and MLE + H_2_O_2_, SWE + ASA + SA + H_2_O_2_ for optimum sowing. Minimum plant height was recorded in unsprayed maize plants in both planting dates (Fig 2).

**Fig 1:** Growth of maize influenced by foliar applied growth promoting agents and sowing dates.

**Fig 2:** Growth of maize influenced by foliar applied growth promoting agents and sowing dates.

### 3.2. Physiological attributes

All foliar applications significantly improved photosynthetic rate while application of SWE + ASA + SA + H_2_O_2_ was found the most efficient and was statistically at par with SWE + ASA, MLE + H_2_O_2_ and followed by ASA + SA + H_2_O_2_. Least photosynthetic rate was examined in control and plants which were sprayed with distilled water. The interaction of sowing dates and foliar application remained non-significant. All foliar applications including distilled water improved transpiration rate however performance of SWE + ASA, MLE + H_2_O_2_ and SWE + ASA + SA + H_2_O_2_ revealed better than others. Minimum transpiration rate was recorded in untreated plants. Highest stomatal conductance was examined in maize plants sprayed with SWE + ASA trailed by SWE + ASA + SA + H_2_O_2_, MLE + H_2_O_2_ and ASA + SA + H_2_O_2_ (Table 1). Lowest stomatal conductance was computed in unsprayed and DWS plants. Data computed for sub stomatal CO_2_ concentration, demonstrated that significantly higher CO_2_ concentration was observed in maize plants sprayed with MLE + H_2_O_2_, SWE + ASA + SA + H_2_O_2_ and found at par with SWE + ASA (Table 1). Lowest CO_2_ concentration was exhibited by unsprayed plants succeeded by distilled water spray. Individual effect of sowing dates and their interaction with foliar applications remained insignificant (Table 1).

**Table 1:** Gaseous exchange attributes of maize influenced by foliar applied growth promoting agents and sowing dates.

Seed Priming	Photosynthesis rate		Transpiration rate		Stomatal conductance		Internal CO_2_ concentration	
	(μmol CO_2_ m^-2^ s^-1^)		(Mmol H_2_O m^-2^ s^-1^)		(Mol m^-2^ s^-1^)		(μmol mol^-1^)	
	S1	S2	S1	S2	S1	S2	S1	S2
**Control**	12.09 f	11.38 f	2.92 d	3.08 d	0.20 de	0.15 e	98.25 d	106.50 d
**Water spray**	14.26 def	14.16 ef	3.47 cd	3.75 bcd	0.18 de	0.21 d	118.75 c	108.00 d
**MLE+H**_**2**_ **O**_**2**_	23.47 a	18.48 bcd	4.70 a	4.90 a	0.29 bc	0.28 bc	167.50 a	164.75 a
**SWE+ASA**	20.12 abc	21.86 ab	5.19 a	4.91 a	0.34 a	0.32 ab	157.00 ab	161.00 ab
**ASA+SA+H**_**2**_ **O**_**2**_	21.60 abc	17.32 cde	4.42 ab	4.36 abc	0.28 bc	0.26 c	152.25 b	158.25 ab
**SWE+ASA+SA+H**_**2**_ **O**_**2**_	23.64 a	22.26 ab	4.70 a	4.79 a	0.31 ab	0.28 bc	160.50 ab	159.75 ab
***LSD at p = 0*.*05 for interaction***	4.47		0.93		0.05		10.68	

S1: Early sowing; S2: Optimum sowing

### 3.3. Biochemical analysis

All foliar applications significantly improved chlorophyll *a* and *b* contents over control and distilled water spray. Highest chlorophyll *a* and *b* activity was examined in SWE + ASA, SWE + ASA + SA + H_2_O_2_ that was statistically like ASA + SA + H_2_O_2_ and MLE + H_2_O_2_. While the lowest chlorophyll contents were computed in DWS and control (Fig 3). Decreased membrane stability index was recorded in unsprayed plants or plants sprayed with distilled water (Fig 3). Higher CAT activity was recorded in plants with the application of SWE + ASA that was statistically at par with SWE + ASA + SA + H_2_O_2_, ASA + SA + H_2_O_2_ in both sowing dates (Fig 4). Highest POD activity was recorded in maize plants that were sprayed with SWE + ASA and found at par with MLE + H_2_O_2_, SW + ASA + SA + H_2_O_2_ followed by ASA + SA + H_2_O_2_ and DWS. Minimum POD activity was examined in control. Highest SOD activity was recorded in SWE + ASA, SWE + ASA + SA + H_2_O_2_ trailed by MLE + H_2_O_2_, ASA + SA + H_2_O_2_ and DWS (Fig 4). Lowest SOD activity was examined in unsprayed and DWS plants. Interaction between sowing dates and foliar application was found insignificant (Fig 4). Maximum phenolic contents were observed in maize plants treated with SWE + ASA chased by SWE + ASA + SA + H_2_O_2_, MLE + H_2_O_2_ or ASA + SA + H_2_O_2_. Minimum phenolics were recorded in DWS and control (Fig 5). Maximum soluble sugars were examined in SWE + ASA chased by SWE + ASA+ SA + H_2_O_2_, MLE + H_2_O_2_ or ASA + SA + H_2_O_2_. Minimum number of soluble sugars was recorded in plants sprayed with distilled water and plants with no treatment sprayed at all (Fig 5).

**Fig 3:** Chlorophyll a, b and membrane stability index of maize influenced by foliar applied growth promoting agents and sowing dates.

**Fig 4:** Antioxidant enzymes of maize influenced by foliar applied growth promoting agents and sowing dates.

**Fig 5:** Phenolic and total soluble sugars of maize influenced by foliar applied growth promoting agents and sowing dates.

### 3.4. Yield and related attributes

Highest numbers of cobs per plant was achieved using SWE + ASA and SWE + ASA + SA + H_2_O_2_ that were was statistically at a similar level with MLE + H_2_O_2_ and then the ASA + SA + H_2_O_2_ as compared to control. Lowest numbers of cobs per plant were recorded in unsprayed plants succeeded by distilled water spray (Table 2). The interaction of sowing dates and foliar applications proved insignificant. Early sowing provided cobs with better diameter than optimal sowing. Greatest cob diameter was recorded in MLE + H_2_O_2_, SWE + ASA and followed by SWE + ASA + SA + H_2_O_2_ or ASA + SA + H_2_O_2_. Lowest cob diameters were linked with control and DWS (Table 2). Comparatively heavier grains were given by recorded in early sowing than optimal sowing. Highest grain weight was linked with the foliar application of SWE + ASA that was statistically at a similar level with MLE + H_2_O_2_ and chased by SWE + ASA + SA + H_2_O_2_ or ASA + SA + H_2_O_2_. Lowest 1000-grains weight was examined in unsprayed maize plants that were statistically similar to DWS (Table 2). Early sowing provided better grain yield over optimum sowing. All foliar applications significantly increased maize grain and biological yields while maximum was observed in SWE + ASA followed by SWE + ASA + SA + H_2_O_2_ or MLE + H_2_O_2_ that were statistically at par with ASA + SA + H_2_O_2_ but plants without spray or distilled water application did not improve grain and biological yields. Minimum maize grain yield was recorded from experimental units of unsprayed plants and succeeded by DWS. The interactive effect of sowing dates and foliar applications were examined insignificant (Table 2). Statistically better biological yield was furnished by early planted maize crop. All foliar applications of growth promoting substances notably improved biological yield of maize and highest was recorded by the application of SWE + ASA that was statistically at a similar level with MLE + H_2_O_2_ or SWE + ASA + SA + H_2_O_2_ and followed by ASA + SA + H_2_O_2_. Lowest biological yield of maize was associated with unsprayed plants and thrived by DWS (Table 2).

**Table 2:** Yield and related attributes of maize influenced by foliar applied growth promoting agents and sowing dates.

Seed Priming	Cobs per plant		Grains per cob		Cob diameter (cm)		1000 grain weight (g)		Grain yield (Mg ha^-1^)		Biological yield (Mg ha^-1^)	
	S1	S2	S1	S2	S1	S2	S1	S2	S1	S2	S1	S2
**Control**	1.15 ef	1.09 f	480.00 de	439.25 f	4.11 def	4.05 f	243.94 cde	224.20 e	4.50 f	4.04 h	13.24 ef	12.98 f
**Water spray**	1.24 cd	1.11 f	491.00 cde	474.25 e	4.12 def	4.07 ef	253.41 abc	232.48 de	4.68 e	4.24 g	13.90 d	13.60 de
**MLE+H**_**2**_ **O**_**2**_	1.32 ab	1.15 ef	550.25 a	510.00 bc	4.32 a	4.25 a	264.21 ab	249.90 a-d	5.90 ab	5.42 d	15.26 ab	14.95 bc
**SWE+ASA**	1.35 a	1.20 cde	550.50 a	530.50 ab	4.30 a	4.21 bc	267.34 a	252.48 abc	6.05 a	5.59 b	15.41 a	15.15 abc
**ASA+SA+H**_**2**_ **O**_**2**_	1.27 bc	1.14 ef	501.00 cd	487.75 de	4.15 cde	4.10 def	244.18 cde	238.47 cde	5.80 b	5.31 d	15.09 abc	14.77 c
**SWE+ASA+SA+H**_**2**_ **O**_**2**_	1.32 ab	1.19 de	537.50 a	510.00 bc	4.17 bcd	4.15 cde	245.75 bcd	239.42 cde	5.89 ab	5.43 cd	15.23 ab	14.93 bc
***LSD at p = 0*.*05 for interaction***	0.06		20.46		0.08		19.99		0.15		0.431	

S1: Early sowing; S2: Optimum sowing.

### 3.5. Principal component analysis

Exogenous application of growth promoting agents and sowing dates significantly influenced the physiological, yield and its related parameters of maize (Fig 6). Parameters (cob diameter, grain per cob and cobs per plant) and (1000-grain weight and grains per cob) shown in quadrant 1 were significantly influenced by T2 (SWE+H_2_O_2_) and T3 (MLE+H_2_O_2_) at early and late sowing dates respectively. Whereas parameters (transpiration rate, stomatal conductance, internal CO_2_ concentration, biological yield, grain yield and photosynthesis rate) shown in quadrant 4 were significantly T4 (ASA+SA+H_2_O_2_ T5 (SWE+ASA+SA+H_2_O_2_) at S1. In addition, parameters (stomatal conductance, transpiration rate, grain yield, photosynthesis rate, internal CO_2_ concentration, biological yield and cobs per plant) were significantly by T4 and T5 at S2. All physiological, yield and related attributes exhibited highest cosine values on F1 axis except grain weight when sown early (S1). Grain weight (early sowing) had highest cosine value at F2-axis with T4. However, GW-S1 and T4 are located in opposite quadrants thus depict the negative correlation among each other.

**Fig 6:** Principal component analysis among foliar applied growth promoting agents, sowing dates and physiological, yield, and related attributes of maize. Clustering of variables has been shown according to highest cosine values on F1 (blue shading) and F2 (red shading). T0: Control; T1: Water spray; T2: SWE+H_2_O_2_; T3: MLE+H2O2; T4: ASA+SA+H_2_O_2_; T5: SWE+ASA+SA+H_2_O_2_; S1: Early sowing; S2: Optimum sowing; CD: Cob diameter; GW: 1000-grain weight; GC: Grains per cob; CP: Cobs per plant; SC: Stomatal conductance; TR: Transpiration rate; ICC: Internal CO_2_ concentration; BY: Biological yield; GY: Grain yield; PR: Photosynthesis rate.

## 4. Discussion

Exogenous application of organic compounds like antioxidants, Osmo protectants and plant growth regulators is being practiced lessening the undesirable effects of environmental stresses in crop plants [11]. It is a cost effective and rapid solution to persuade abiotic stress forbearance in plants such as chilling, heat, drought and salinity [22]. The following study was aimed for the improvement of the thermotolerance of the spring maize by using the foliar application of growth promoting substances at critical growth stages under early and optimum sowing dates. The results obtained are similar to many researchers who have observed the positive effects of these growth promoting substances when applied exogenously to different crops. Janda et al. [23] reported that exogenous application of SA improved chilling tolerance in maize, H_2_O_2_ in wheat [18] and ASA in wheat [17]. Yasmeen et al. [14, 15] concluded that exogenous application of MLE promoted abiotic stress tolerance, growth, and yield in wheat under stressed conditions.

An infrequent increase in maize growing pattern was observed by the exogenous application. Net assimilation rate, crop growth rate and dry matter accumulation were seen to be enhanced by the exogenous application of growth promoting substances (Fig 1). The impact of highly vigorous crop growth was the result of such application and affected photosynthetic activities and leaf area duration, positively to the maximum levels. As a result, high accumulation of assimilates in grains were recorded [25, 26]. It was observed that MLE can stimulate hormones like cytokinin to form and prevent premature leaf senescence, causing larger leaf area with higher accumulation of photosynthetic pigments [27, 28]. Rapid cell division is influenced due to availability of hormones for plants, antioxidants, phenolics, minerals in the solutions used as foliar sprays. SWE was reported by Dykes and Rooney [28] as a good source tannins, flavonoids and phenolic acids. The alkaloids confined in the SWE are the pioneers of the regulators of growth and are highly engaged in plant’s defense mechanism against various stresses [29]. MLE holds substantial amounts of cytokinin in the shape of antioxidants, ascorbates, and phenols along with abundant potassium and calcium [30]. The increase in dry matter accumulation and crop growth rate is mainly due to the foliar application of ascorbic acid, salicylic acid and H_2_O_2_ which increases the cell division and protects the chlorophyll and membranes present in the cells. Many researchers found that low concentrations of SA had positive influence on maize growth [31–33], whereas high concentrations provoked inhibitory effects [34]. These results are in line with the findings of other researchers who found improvement in dry mass with exogenous application of SA in maize [35], ASA in wheat [36] and H_2_O_2_ in wheat under stressed conditions [18, 37].

Substantial increase in photosynthetic and transpiration rates along with stomatal conductance and internal CO_2_ concentration of treated plants (Table 1) was due to enhanced antioxidant enzyme activities, better photosynthetic pigments, and elevated resistance to temperature extremes. Though all foliar applications proved effective in boosting physiological performance of the crop, but maximum values of these attributes were linked with MLE + H_2_O_2_, SWE + ASA and SWE + ASA + SA + H_2_O_2_. As SWE and MLE are rich in growth promoting substances, they showed maximum improvement in all attributes along with other synthetic growth enhancers. It is found that applying SA will promote photosynthetic pigments and photosynthesis rate in maize [38, 39]. Exogenously applied SA was found positive on growth, photosynthesis and is also responsible for tolerance in stress conditions of the plants [31, 40, 41]. The physiological processes of a plant that includes economic yield, seed germination, transpiration rate stomatal conductance and photosynthesis can be highly influenced by the application of SA [42]. High periodic activity was observed in maize plants that were treated by the growth promoting agents, which resultantly led to better crop and growth development of the maize.

Enhanced leaf senescence due to the heat stress causes a decrease in chlorophyll amount hence, lower leaf area duration and photosynthesis [43]. It was recorded that all the exogenous applications substantially increased the chlorophyll contents during both, early and optimum sowing dates. However, the plants with no application of growth promoting substances showed poor results (Fig 3). It is reported that high temperature at early growth stages enhances crop growth due to increase in chlorophyll activity and crop grows vigorously. But at the later stages of development, the process of leaf senescence started under temperature stress conditions resulting in the loss or degradation of chlorophyll. Spano et al. [44] declared that active period dedicated to photosynthesis can improve total photosynthates available in the life of the crop. Higher mass of each grain can be obtained achieved if maintenance regarding the assimilated levels of carbon to grains through the process of grain filling period. The winter crop species of cereals experiences turning down of chlorophyll contents due to heat stress, and this dismissal of chlorophyll leads to many physiological damages [45]. Obtained results are in accordance with those of Sakr and Arafa [46] who showed that chlorophyll contents were increased in canola when antioxidants were applied to the plants under salinity stress. Exogenously applied hydrogen peroxide, ascorbic acid and salicylic acid successfully increased chlorophyll a and b in maize [38], wheat [18, 47], respectively under stressful conditions. Exogeneous application of growth promoting agents also enhances the cell membrane stability of a plant (Fig 3). Like other growth enhancers, exogenous application of MLE also considerably improved cell membrane stability. MLE is a natural source of cytokinin and nutrients especially potassium which plays important role in osmotic adjustment during stressful environment [24]. Applying cytokinin under heat stress can increase membrane stability, chlorophyll contents and grain yield of wheat [48].

Significant correlation of cell antioxidants and temperature stress tolerance has been concluded by many researchers [49]. Reactive oxygen species (ROS) production is the response of different oxidative stresses which includes high temperatures and causes damage to proteins, nucleic acids and lipids, of the plant systems. The ROS are eliminated by antioxidant compounds and enzymes [50], while higher temperatures can be a reason of reducing the activities of POD, SOD and CAT [28]. Under stressful conditions, the antioxidant system of the plants is not strong enough to reduce the injuries of oxidative stress. So, crop plants are in need of some external assistance to cope with this abiotic mischief. All exogenous application of growth promoting substances significantly improved CAT, POD, SOD activities including phenolics (Fig 4). However, maximum improvement in antioxidant defense system was observed in combinations containing SWE and MLE. SWE is rich in phenolic compounds which includes phenolic acids [51, 52] and sorgoleone [53–55]. Phenolics are secondary metabolites, which are produced when plants undergo stressed conditions and helps to protect cell structures from injuries caused by oxidative damage [56].

Phenolics being the powerful antioxidants of the plants, have a pivotal role in plant defense against abiotic stressors [57]. Phenolic tolerate abiotic stress by scavenging of free radicals produced under stressed conditions and performs a number of functions in the plant [58]. Siddhuraju and Becker [59, 60] reported that MLE is an excellent natural source of antioxidants like phenolics which performs their scavenging actions during stressed conditions. It was reported that the antioxidant enzymes increased their activity when the ascorbic acid and salicylic acid was applied exogenously, under drought and salt stress conditions, respectively [17, 36]. Whereas H_2_O_2_ also showed positive results when different stresses were induced in wheat [18, 61]. Total soluble sugars are categorized as plant primary metabolites and primary metabolites are involved in osmotic adjustments when the formation of cell structures takes place [62]. Exogenous application of growth enhancing agent’s considerably improved total soluble sugars in maize leaves under both sowing conditions. Comparatively higher soluble sugars were recorded in early sowing and performance of SWE+ASA was found superior in both planting dates (Fig 5). It is reported that under various environmental stresses, sugars are accumulated in crop plants [63]. The mobilization of sugars in various parts of the plants is affected by environmental factors such as heat stress and salinity [64].

Yield contributing characters attributes are the most important factors that directly contributes towards the economic yield of the grain. That has direct contribution towards economic yield. Higher temperatures stress reduced the number of grains per cob and weight of grain of plants ever controlled in both sowings. Via the foliar use of substances that encourage growth the yield of grain was increased and its attributes under each sowing date but most betterment was seen in early sowing. This might be the impact of early crop growth and development in initially grown crop. The units of maize that were planted early showed a higher performance in almost every attribute. Highest biological and grain yields were as observed by foliar application of SWE + ASA and MLE + H_2_O_2_ (Table 2). Obtained results are par with Jabran et al. [65] who found that the foliar applications of SWE increased the yield of wheat. In another study, Cheema and Khaliq [66] concluded that two sprays of SWE on wheat can increase the yield up to 20%. ASA also contributed equally with SWE and played critical role in boosting maize growth and yield. Barth et al. [67] reported that ASA is an essential co-factor in plant hormones synthesis process. Furthermore, the application of exogenous ASA has shown to improve the mitotic activity in maize [68, 69].

## 5. Conclusion

The enhanced grain yield and crop performance under extreme temperature stress can be achieved by treating maize seedlings with different growth promoting agents. The following study monitored the effects of some natural and artificial growth promoting substances. Among different combinations of natural and synthetic growth promoting agents, SWE + ASA, MLE + H_2_O_2_ and SWE + ASA + SA + H_2_O_2_ were the best combinations for improving growth, development, and physiological variables under both sowing dates even under suboptimal temperature. Enhanced maize grain and biological yields were observed in SWE + ASA followed by SWE + ASA + SA + H_2_O_2_ or MLE + H_2_O_2_ that were statistically at par with ASA + SA + H_2_O_2_ but plants without spray or distilled water application did not improve grain and biological yields The result of current study stated that SWE + ASA, MLE + H_2_O_2_ and SWE + ASA + SA + H_2_O_2_ showed the best results among all other foliar applied combinations. Taking together, these combinations proved beneficial to enhance maize crop growth, development, yield, and biochemical variables during high temperature stress under early and optimum sowing dates.
